# A Probe into the Counterfeiting of Academic Journals from Multiple Player Perspective

This article has been retracted.

**DOI:** 10.1155/2022/3054668

**Published:** 2022-05-21

**Authors:** Ai Lei, Chuhan Qian

**Affiliations:** School of Information Management, Nanjing University, Nanjing 210023, China

## Abstract

Scholars have been suffering from scams involving counterfeit academic journals for a long time, and there has been a relatively clear analysis of the causes of counterfeiting and the governance path for it in existing studies. However, the authors reexamined the counterfeiting and found the problem still prevails. Through the analysis of the multiple players involved in counterfeiting, the author points out that the current personnel evaluation mechanism and journal evaluation system are the root causes of counterfeiting and thus offer corresponding suggestions for further improvement.

## 1. Introduction

As information technology improves by leaps and bounds in China, the digital transformation of academic journals has failed to meet the authors' needs for paper contribution. This provides an opportunity for lawbreakers to counterfeit academic journal websites or submission websites, or send emails to authors to invite contributions in the name of the editorial department of a specific academic journal to cheat the authors of their money. During China's crackdown against pornography and illegal publications from 2010 to 2018, the cases of counterfeiting academic journals had been ranked among the top 10 each year [1]. In contrast, they did not appear on the top 10 lists from 2019 to 2021, but the author's investigation reveals that the counterfeiting problem becomes even more serious. This study is aimed to identify the institutional roots of counterfeiting and propose possible resolutions to this die-hard social problem based on the analysis of the current situation of counterfeiting and the players involved in it.

## 2. Current Research on the Counterfeiting of Academic Journals

The research on the counterfeiting of academic journals by Chinese scholars began in 1998 when Zhang Zhiqing investigated the activities of counterfeiting academic journals for fraudulent purposes. The research then focused on activities such as the fraudulent publication of fake academic journals by unscrupulous people, and Zhang's opinion on such phenomenon was to strengthen regulations and legal crackdowns [2]. The research from 1999 to 2010 mainly focused on the study and governance of illegal journals. With the emergence of large-scale applications in the Internet era, since 2011, the academic community has focused on the counterfeiting of academic journal websites. In these studies, fake submission websites, “phishing emails,” and other fraudulent ways of counterfeiting academic journals were also mentioned, and the research reached a minor peak in 2016 [3–5]. In December of the same year, under the deployment of the National Office for National Office Against Pornographic and Illegal Publication and the former State Administration of Press, Publication, Radio, Film and Television, the local offices against Pornographic and Illegal Publications took the lead to carry out a special crackdown and rectification on such illegal activities, especially the counterfeiting of academic journal websites [6]. Since 2018, studies have been conducted from the perspectives of criminal justice, empirical search engine, governance of different platforms, multidimensional perspectives, and different disciplines. Meanwhile, some journals have also given advice publicly on how it “outwit” fraudsters to help authors protect their rights and recover losses, but it is an exception. The current study focuses on the description of the phenomenon, the explanation of the causes, and proposed strategies to deal with this issue. It basically clarifies the responsibilities of five related subjects such as authors, academic journals, regulatory authorities, search engines, and judicial departments [7–12].

Existing studies suggest that several factors contribute to the counterfeiting of academic journals. First, at the authors' level, they lack awareness and professional ethics, so they should raise their security awareness and promptly defend their rights after being cheated. Second, at the academic journals' level, their information channels for contribution are not wide enough and they fail to speak out in time when faced with counterfeiting and lack the power to protect their rights. Therefore, academic journals should broaden the information channel to increase recognition, appeal to the regulatory authorities in conjunction with industry associations, and negotiate with search engines for solutions. Third, search engine service providers should fulfill their main responsibility to strengthen the audits that were neglected earlier for the sake of profit. Fourth, the regulatory authorities should establish a sound supervision reporting mechanism while the judicial departments should increase the legislation and sentencing for such crimes [7–12].

A search for “counterfeit academic journal website” on the *Web of Science* found only one relevant article, and it was written by a Chinese scholar from Jinan University who studied such issues in China. Wang Xiaofei et al. pointed out that foreign academic journals are normally published online by several major publishing groups for free, which would be handled by professionals uniformly in case of copyright infringement. That's why few foreign academic journal websites are being counterfeited [13].

To sum up, existing researches have disassembled the occurrence links of counterfeiting of academic journals and proposed specific methods for relevant players' improvement. However, the author's investigations between August and September 2021, show that the situation has not been improved while scams in various forms are still rampant and scammers are even able to avoid legal risks, which put higher demands on the personal integrity and recognition ability of the paper authors.

## 3. Investigation and Causes of Counterfeiting of Academic Journals in Recent Five Years

### 3.1. The Counterfeiting of Academic Journals Remains Serious

As mentioned above, the national special crackdown on counterfeit academic journals was carried out in December 2016. Then the author searched the keyword “statement on counterfeiting” on CNKI (Chinese mainstream knowledge service website). Between January 2017 and July 26, 2021, a total of 361 journals issued warnings on counterfeit websites, covering a wide range of disciplines including medicine and social sciences, as shown in Figure 1.

In recent years, “core/authoritative/source journals” have been introduced by various institutions into their personnel evaluation system as a decisive basis for assessing their staff's degrees, employment, professional titles, awards, projects, and ranks [13]). The professional titles of many practitioners, such as teachers and doctors, depend much on the publication of the papers too. As a result, the paper publication has become the most immediate need for many people. Actually, the mismatch between the limited number of high-quality academic journals and the great demand for the publication of papers results in fraud.

Figure 1 shows that journals of most disciplines have been counterfeited, precisely because the institutions involving these disciplines have made the number of published papers a decisive factor to determine their staff's performance appraisal, title evaluation, and promotion, resulting in a large demand for paper publication. Medical and educational journals are the ones that account for the highest percentages because personnel engaged in these substantive disciplines are required to have a considerable number of papers published for appraisal or promotion. However, these people, who are more practitioners than academics, are vulnerable to scams of counterfeiting since they are not quite familiar with academic journals.

### 3.2. Diversified and More Blurred Forms of Fraud

The counterfeit journals were “advancing with the times” by creating various channels in all corners of the Internet, ranging from their official websites to search engines to contacts on QQ, WeChat, and even mini-programs. Scammers took advantage of the author's eagerness to publish the paper and set up stores for “phishing” on shopping websites. The “service for publishing papers” became a standardized product on such websites. Search by the keyword “papers” on Taobao, Pinduoduo, and other mainstream shopping websites, and you will see a flood of information about the publication of papers, pop-up details suggesting that the papers have to be reviewed, and published quickly by the core journals recognized by authoritative institutions. As early as 2015, seven departments [14] jointly issued a “Five Prohibitions” on the publication of academic papers, one of which prohibited “the third parties” from submitting papers on behalf of the authors.

However, the author found more than 3,600 related services when searching the keywords “paper” and “contribution” on major shopping websites such as Taobao and Pindoduo. After combing and deduplicating the search results, we obtained the word cloud map displaying service titles as shown in Figure 2. It can be found from Figure 2 that even “ghostwriting,” the act of writing papers for others, has appeared on shopping websites; and medical care, finance, and teachers are still hot words indicating the strong market demand for the publication of papers in these disciplines. The author contacted the store with the highest number of transactions, and the customer service representative requested all communications to be made through WeChat for “one-to-one” services. The avatar of the representative on Wechat was a professionally dressed woman, which easily wins people's trust. She claimed that she could get papers published in the core journals recognized by China's academic community once the deposit payment was made. Meanwhile, this WeChat customer service representative gave the names of many academic journals with whom they have been in cooperation and showed some examples of their “successful” cases, which would make her business seem more reliable. However, such a transaction process has been moved beyond the shopping platform, so even if the paper ends up not being published, it is impossible to get the deposit back. Such scams in the disguise of a trading dispute on the platform are more difficult to identify and handle.

### 3.3. Slow Informatization Improvement of Academic Journals

Based on an in-depth analysis of the five players involved in the existing research, it can be found that the academic journals are at the core of solving the problem. Search engines and regulatory authorities are mostly passive in their actions because there is massive information on the Internet that needs to be reviewed and monitored. The judicial department needs a long-term judicial practice before making any adjustment to the current process. Furthermore, due to the low cost of counterfeiting, lawbreakers can set up multiple fake websites at the same time and replace a batch after a while. From the author's point of view, each year they will see new members join the profession or the academic community with an evaluation mechanism requiring the publication of papers That's why the new members will have an urge to get their papers published but it takes time for them to develop information literacy and security awareness.

From the perspective of academic journals, they will exist for a long time once they are established. Even though the editorial department is not powerful enough to help the deceived authors protect their rights, it is the general trend to actively promote the information construction for the development of academic journals in the digital era. Therefore, it can be said that academic journals are at the core of solving such problems.

Take the Chinese social science journals, for example. The author randomly selected 200 journals from the CSSCI catalog for 2019–2020 and found that a total of 40 journals had issued a notice about “statement on counterfeiting” in the past 3 years, which means the proportion of counterfeiting is 20%. After keying in the names of the above-mentioned counterfeited academic journals on search engines, we found that the top web pages were still those counterfeit websites claiming rapid publication of papers, and the authors were still very likely to be cheated.

Through the analysis of the above-mentioned statements on counterfeiting, we found that the statements simply warned the authors against scams while presenting the proper way for paper contribution. Only *Management World* stated that it would actively take legal action to protect its rights and interests. In the case of being counterfeited, the concerned journals merely published a statement but did not take relevant actions such as reporting to the police or filing a lawsuit, which was of little deterrence against lawbreakers. This also explains why counterfeiting keeps perpetuating.

Theoretically, it is believed that the academic journals being counterfeited should pay more attention to establishing sound communication channels with authors. The authors investigated the 40 journals being counterfeited about their WeChat official accounts (WOA), the registration subjects of WOAs, whether the WOAs have the function of checking manuscripts, and whether they have direct channels for paper submission on CNKI. The results are shown in Table 1.

The results showed that most of the academic journals being counterfeited did not take active action to establish information channels with authors. Although they opened WOA, the account's subjects either did not go through official certification or did not improve the function of notification for paper contribution. In particular, many academic journals have not set up a submission channel on CNKI that is more familiar to authors. In fact, many academic journals did not take active improvement measures even after being counterfeited.

### 3.4. Roots-Personnel Evaluation Mechanism and Academic Journal Evaluation System

Existing studies have mentioned that the counterfeiting of an academic journal can have a negative impact on the reputation of the journal itself. However, Figure 3 shows that the composite impact factors of these 40 academic journals in the last 4 years from 2017 to 2020, showed that the 27 journals, for which data were available, were seen with an increasing trend in both the composite and compound impact factors. It indicated that a negative impact on the reputation of academic journals did not mean that authors were less willing to contribute papers to the journal. The journals were not losing good authors and high-quality papers.

The results showed that the most critical evaluation indexes for academic journals, namely, composite and compound impact factors, were on an upward trend even if the journals had been counterfeited, and the evaluation standard impact factor of academic journals was not based on the smoothness of submission channels. The counterfeiting did not cause substantial damage to the academic journals. As a result, these journals did not pay enough attention to the problem, without holding the search engines liable for counterfeiting or reporting to the competent authorities for solutions, and thus counterfeiting remained widespread and seriously affected the academic ecology.

In terms of the social division of labor, authors are producers of knowledge, whereas academic journals are disseminators of knowledge. The two parties share symbiotic interests in the academic community. However, their respective evaluation systems make them conflict with each other. Some authors try all means to get their papers published because a considerable number of institutions emphasize the quantity and quality of the published papers when appraising their staff. As pointed out by Xi Zhiwu, most of the deceived authors are young scholars with insufficient information literacy and lack of experience in paper submission, making them easy targets for scams. On the other hand, to maintain their influence, academic journals contact the head institutions and head authors who produce high-quality papers, which is an important guarantee for the influence of academic journals [13]). From the 1970s, when the theoretical studies emerged, to the present, the evaluation of academic journals has been gradually localized, diversified, and integrated, and the four major evaluation bodies now have strong credibility and have contributed greatly to the optimization of the academic environment. Yet journal evaluation has been inappropriately assigned the role of determining the evaluation of scholarly output.

Therefore, the roots of the current fraud lie in the current personnel evaluation system based on the publication of papers and the evaluation system for academic journals based on quantitative impact factors.

## 4. Suggestions for Governing the Counterfeiting of Academic Journals

In his speech at the symposium for scientists, General Secretary Xi Jinping clearly pointed out the need to run first-class academic journals and various academic platforms, and to strengthen domestic and international academic exchanges. In June 2021, the Propaganda Department of the CPC Central Committee, the Ministry of Education, and the Ministry of Science and Technology jointly issued a notice on “Opinions on Promoting the Prosperity and Development of Academic Journals,” stating that academic journals are an important platform for academic research and communication, an important position for spreading ideas and culture, and an important factor in the promotion of theoretical innovation and scientific and technological progress; and at the same time, they also proposed to crack down illegal activities such as the counterfeiting of academic journals and their websites. As the pillars of academic system construction, academic journals play an important role in national academic development and innovation.

At the national governance level, the crackdown on illegal activities such as the counterfeiting of academic journals and their websites should be accompanied by a review of the nature and sentencing of such crimes. In his preface to the *Illegal Publishing Activities*, Liu Gao, former deputy director of the State Press and Publication Administration, commented on the judicial department's proposal to address the criminal activities of illegal publications, including the counterfeiting of academic journals [13]. Through the analysis of counterfeiting cases over the past 10 years, Wang Yong pointed out that counterfeiting cases are still punishable by the crime of illegal business rather than the crime of fraud, and there is a large difference in the entrenching between the two. The counterfeiting of academic journals and websites is considered as online scams, and currently, China intends to launch a special Internet Fraud Act dealing with such online criminal activities.

At the evaluation system level, the current rigid personnel evaluation mechanism should be changed. In October 2020, the Central Committee of the CPC and the State Council issued the “General Plan for Deepening Education Evaluation Reform in a New Era,” making a series of new deployments to “Break the Five ” and other new deployments to improve the diversified academic evaluation system by adopting categorical evaluation methods for the diversity and specificity of different disciplines, fields, and job series. It is the general trend to abolish the paper publication as the core of the evaluation system, which is conducive to fundamentally stimulating the internal driving force of talent innovation and academic development. Universities and research institutions attach great importance to the quantitative index of papers when appraising a scholar to objectively evaluate the academic ability of the scholar, stimulate their potential, and promote the benign development of academic ecology. However, the current evaluation and reward system for all kinds of personnel is highly bound to the evaluation of academic journals.

At the level of academic journals' construction, the journals are aimed to serve academia and society. On the one hand, academic journals, as the target of being counterfeited, should not only issue a statement on counterfeiting but also ensure the smooth information channels of the journals. That is, they should establish official websites, open certified official WOAS, improve their visibility on various academic platforms, and set up direct submission links on common academic websites, such as CNKI, to ensure a clear and unambiguous contribution message for authors in the first place. On the other hand, they can entrust a third-party legal defense agency to defend their rights when being counterfeited, and share the proceeds with the agency. This can greatly reduce the cost of defending their rights.

In terms of contributors' personal qualities, those who were cheated are basically academic newcomers or practical workers who do not often write papers or do so only for elevating their titles. First, contributors should improve their information literacy, understand the common academic information and communication platforms, and have the basic ability to distinguish between real and fake academic journal websites; second, they should abide by the code of ethics for academic research with a good attitude and stop taking chances. Furthermore, any contributor being cheated should call the police at the earliest to keep more people from the scam.

In a short term, it is necessary to promote the self-improvement of each body involved in the counterfeiting. In the long run, it is necessary to bring a fundamental improvement in the evaluation system of academic journals, adjust the evaluation mechanism for relevant personnel, rebuild a good social order, and resume the role of papers as academic achievements.

## Figures and Tables

**Figure 1:** Distribution of disciplines for journals issuing “statement on counterfeiting” from January 2017 to July 26, 2021.

**Figure 2:** Word cloud analysis on Taobao's service for ghostwriting and cheating publication of papers.

**Figure 3:** Trends for compound impact factors of 27 academic journals being counterfeited from 2017 to 2020.

**Table 1:** Investigation results of digitalization of journals being counterfeited.

No.	Journal name	Year					
		Discipline	Availability of WOA	Name of WOA	Submission/checking information on WOA (including the link)	Registration subjects of WOA	Submission channel on CNKI
1	Confucius Studies	Philosophy	Yes	Journal of Confucius Studies	N/A	Editorial Department of Confucius Studies	Yes
2	Chinese Linguistics		Yes	Chinese Linguistics	Yes	Personal	Yes
3	Linguistic Researches	Linguistics	Yes	Editorial Department of Linguistic Researches	Yes	Personal	N/A
4	Language Teaching And Linguistic Studies		Yes	Language Teaching And Linguistic Studies	Yes	Personal	Yes
5	Foreign Literature Studies	Foreign literature	Yes	Foreign Literature Studies	Yes	Central China Normal University	N/A
6	Journal of Ming-Qing Fiction Studies		Yes	Journal of Ming-Qing Fiction Studies	Yes	Personal	N/A
7	Historical Studies of Modern Literature	Chinese literature	Yes	Journal of Historical Studies of Modern Literature	N/A	The Editorial Department of Historical Studies of Modern Literature	N/A
8	Comparative Literature in China		Yes	Journal of Comparative Literature in China	Yes	上海外国语大学 Shanghai International Studies University	N/A
9	Journal of Beijing Film Academy	Archology	Yes	Journal of Beijing Film Academy	Yes	*Journal of Beijing Film Academy*	N/A
10	Journal of Beijing Dance Academy		Yes	Journal of Beijing Dance Academy	Yes	The Editorial Department of Journal of Beijing Dance Academy	Yes
11	Musicology in China		Yes	Institute of Music of Chinese National Academy of Arts	Yes	Chinese National Academy of Arts	N/A
12	Art and Design		Yes	Journal of *Art and Design*	Yes	Tsinghua University	Yes
13	Historical Review	History	Yes	Editorial Department of *Historical Review*	Yes	Institute of History, Shanghai Academy of Social Sciences	Yes
14	International Economics and Trade Research		Yes	International Economics and Trade Research	Yes	Guangdong University of Foreign Studies	Yes
15	Intertrade		Yes	Journal of Intertrade	Yes	China Commerce and Trade Press Co., Ltd.	N/A
16	Journal of Financial Research		Yes	Journal of Financial Research	Yes	The journal Office *of Financial Research Co., Ltd.*	N/A
17	Economic Review Journal	Economics	Yes	The office of Economic Review Journal	Yes	The office of *Economic Review Journal*	Yes
18	Journal of Agrotechnical Economics		Yes	Agricultural Economy of China	Yes	China Agricultural Economics Association	Yes
19	Commercial Research		Yes	*Commercial Research*	Yes	The office of *Commercial Research*	Yes
20	Securities Market Herald		Yes	Research of Shenzhen Stock Exchange	Yes	Shenzhen Stock Exchange	Yes
21	Modern Law Science	Law	Yes	Modern Law Science	Yes	Southwest University of Political Science and Law	Yes
22	Peking University Law Journal		Yes	Editorial Department of Peking University Law Journal	N/A	Personal	Yes
23	Folklore Studies		Yes	Folklore Studies	N/A	Personal	N/A
24	Journal of South-Central University for Nationalities (Humanities and Social Sciences)	Ethnology and culturology	Yes	Journal of South-Central University for Nationalities (Humanities and Social Sciences)	Yes	South-Central University for Nationalities	有 yes
25	Science-Technology and Publication	Journalism and communication	Yes	Science-Technology and Publication	Yes	The Office of Science-Technology & *Publication*	N/A
26	Journalism Research		Yes	Journalism Research	Yes	Fudan University	N/A
27	Document, Information and Knowledge	Library, information and philology	Yes	Document, Information and Knowledge	Yes	Personal	N/A
28	Peking University Education Review		Yes	Peking University Education Review	Yes	Peking University	N/A
29	Comparative Education Review	Pedagogy	Yes	Comparative Education Review	Yes	Beijing Normal University	Yes
30	Teacher Education Research		Yes	Teacher Education Research	Yes	Beijing Normal University	Yes
31	Research in Educational Development		Yes	Research in Educational Development	Yes	Shanghai Institute of Educational Sciences	N/A
32	Journal of Educational Studies		Yes	Journal of Educational Studies	Yes	Beijing Normal University	Yes
33	Modern Educational Technology		Yes	Journal of Modern Educational Technology	Yes	Shenzhen International Graduate School of Tsinghua University	Yes
34	Hebei Academic Journal		Yes	Hebei Academic Journal	Yes	The Office of *Hebei Academic Journal*	N/A
35	Seeker	Comprehensive social science	Yes	Journal of Seeker	Yes	Hunan Academy of Social Sciences	Yes
36	Social Science Journal		Yes	Social Science Journal	Yes	Liaoning Academy of Social Sciences	N/A
37	City Planning Review	Human and economic geography	Yes	City Planning Review	Yes	*City Planning Review* Journal Office Co., Ltd.	Yes
38	Journal of Shandong Normal University (Humanities and Social Sciences)	Journal of higher education	Yes	Journal of Shandong Normal University	Yes	Shandong Normal University	N/A
39	Journal of Tongji University (Social Science Section)		Yes	Journal of Tongji University(Social Science Section)	Yes	Tongji University	N/A
40	Journal of Xiamen University (A Quarterly for Studies in Arts and Social Sciences)		Yes	Journal of Xiamen University (A Quarterly for Studies in Arts and Social Sciences)	Yes	Personal	Yes

## Data Availability

We do not have permission to share data from the data provider.
